This article has been retracted.

# Effect of Hysteroscopic Polypectomy Combined with Mirena Placement on Postoperative Adverse Reactions and Recurrence Rate of Endometrial Polyps: Based on a Large-Sample, Single-Center, Retrospective Cohort Study

**DOI:** 10.1155/2022/1232495

**Published:** 2022-04-26

**Authors:** Yanli Shen, Wenguang Feng, Jing Yang, Jinling Yi

**Affiliations:** The Fifth Affiliated Hospital of Xinjiang Medical University, 830011, China

## Abstract

**Objective:**

To investigate the effect of hysteroscopy surgery combined with Mirena on postoperative adverse reactions and recurrence rate of endometrial polyps (EP).

**Methods:**

A total of 312 patients who underwent hysteroscopic polypectomy of EP in our hospital from June 2017 to November 2020 were enrolled retrospectively. Among them, 42 patients did not take any treatment after the operation (control group), 156 patients were treated with levonorgestrel intrauterine birth control system (Mirena group), and 114 patients were treated with oral spironolone ethinylestradiol tablets (oral group). The clinical data of 312 patients were recorded and followed up regularly. All patients were followed up through an outpatient clinic or telephone to 12 months after the operation. The patients' age, disease course, number of pregnancies, clinical manifestations, endometrial thickness before the operation, duration of operation, amount of bleeding during the operation, and number and size of polyps were analyzed. The recurrence and postoperative side effects of EP in the three groups were followed up within 12 months after the operation.

**Results:**

There was no significant difference in endometrial thickness among the three groups before treatment (*P* > 0.05). After 3 months, 6 months, and 12 months of treatment, the endometrial thickness of the three groups decreased, while the decrease in the Mirena group and the oral group was better compared to the control (*P* < 0.05). The decrease in the Mirena group was better than that in the oral group (*P* < 0.05). There was no significant difference in hemoglobin levels among the three groups before treatment (*P* > 0.05). After 3, 6, and 12 months of treatment, the hemoglobin levels of the three groups increased to varying degrees, while the levels of the Mirena group and oral group were better compared to the control (*P* < 0.05). Three months after the operation, the improvement of clinical symptoms was similar in the three groups, and there was no significant difference among the three groups (*P* > 0.05). At 6 and 12 months after the operation, the improvement of clinical symptoms in the oral group and Mirena group was better compared to the control group (*P* < 0.05), but there was no significant difference between the oral group and Mirena group (*P* > 0.05). After the operation, some patients had complications such as lower abdominal pain, breast distension pain, irregular vaginal bleeding, and abnormal liver function. There was no significant difference in the number of complications among the three groups (*P* > 0.05). During the follow-up to 12 months after the operation, the recurrence rate in the oral group and Mirena group was lower compared to the control (*P* < 0.05), and the recurrence rate in the Mirena group was lower than that in the oral group (*P* < 0.05).

**Conclusion:**

Placing Mirena immediately after hysteroscopic polypectomy of EP can reduce the recurrence rate of endometrial polyps, increase the level of hemoglobin, and reduce the thickness of the endometrium, which can be employed and popularized according to the condition of patients in clinical work.

## 1. Introduction

Endometrial polyps (EP) are induced by local overgrowth of endometrial tissue, which is composed of different numbers of glands, stroma, and blood vessels covered by epithelium [1]. The matrix of polyps consists of fibroblast-like fusiform cells and thick-walled large blood vessels. The premenopausal polyp epithelium may be active and pseudostratified, and after menopause, it may become inactive and flat [2]. EP can occur in females of any age and is common in females of childbearing age. They may appear in single or multiple forms, may be sessile or pedicled, and range in size from millimeters to centimeters [1, 2]. In addition to glands and stroma, EP also includes smooth muscle fibers, called adenomatous polyps [3]. Up to now, the etiology of EP is not clear [4], as one of the very common gynecological diseases, because there is no particularity of clinical manifestations and it is easy to misdiagnosis and delay the diagnosis, so the exact prevalence rate is difficult to estimate, perhaps 7.8% to 34.9%, depending on the population studied [5]. EP mainly occurs in women over 35 years old, especially in women approximately 50 years old. The clinical symptom of endometrial polyps is mainly menstrual changes, often manifested as abnormal uterine bleeding [6], including infertility, but there are still some patients without any clinical symptoms [7]. Transvaginal ultrasound (TVUS) is the primary choice for the examination of endometrial polyps, and TVUS is more accurate during the proliferative phase of the menstrual cycle [8]. For the patients with high intrauterine echo and endometrial thickness > 8 cm by transvaginal ultrasound, hysteroscopy and biopsy are recommended. At present, the treatment methods for endometrial polyps are as follows: (1) observation and waiting: suitable for asymptomatic and polyp diameter < 1 cm [9, 10]; (2) progesterone drug therapy; and (3) surgery: in patients with polyp diameter > 1 cm and obvious clinical symptoms, polyp removal and diagnostic curettage can be performed; endometrial ablation can be recommended for patients with no fertility requirements and recurrent; hysterectomy can be considered for those with malignant tendency [11–13]. Surgical treatment is mainly used for patients with clinical symptoms. Hysteroscopic polypectomy is the first choice for the diagnosis and treatment of EP. However, in clinical work, it is found that most patients are easy to relapse after simple surgical resection and come to see a doctor with the same symptoms again [13]. The recurrence rate after EP is high, which has increased to 9.38% in recent years [14]. Finding an effective treatment to reduce the recurrence rate of EP is the main problem in the current clinical duties.

It is urgent to seek effective treatment to restrain the recurrence of EP, reduce the rate of rehospitalization and operation, and decrease the cost of health insurance [14]. Due to the physiological effects of estrogen and progesterone, some studies [15–17] have shown that EP is an estrogen-dependent disease, and its pathogenesis is related to the high level of estrogen in the body. Progesterone can transform the endometrium to the secretory phase on the basis of estrogen [16]. Li et al. and other studies found that progesterone could slow down the recurrence of endometrial polyps [18]. However, long-term systemic use of hormone drugs has side effects and inconvenience, and many patients lack compliance. Therefore, it is necessary to develop some new drugs or ways that can reduce the recurrence of EP to improve the quality of life of patients.

Levonorgestrel intrauterine birth control system (LNG-1US, Mirena) is an efficient, safe, long-term, and reversible IUD. This kind of IUD has the advantages of reducing menstrual volume and relieving dysmenorrhea. Levonorgestrel contains levonorgestrel. The effect of local controlled release of progesterone may be equivalent to or even better than that of oral progesterone [19]. For example, Ying's study found that LNG-IUS for patients with adenomyosis could significantly relieve dysmenorrhea, reduce menstrual blood, decrease uterine volume, and increase the content of hemoglobin; for patients with dysfunctional uterine bleeding, while reducing the amount of menstruation, the endometrial shedding and thinning, the menstrual period gradually shortened with the extension of placement time, endometrial proliferative lesions can be cured [19]. Compared with ordinary progesterone, Mirena has better advantages such as follows: (1) the adverse reactions of its own systems are reduced to avoid low levels of estrogen; (2) reversible excision has little effect on the long-term pregnancy rates and no reports of fetal malformations; (3) long-term and economical; and (4) it is safe, reliable, and highly tolerable. Mirena has no significant effect on liver and kidney functions. Thus, the purpose of this study is to explore the therapeutic effect of Mirena after hysteroscopic polypectomy of EP and the effect on the postoperative adverse reactions and recurrence rate of EP.

## 2. Patients and Methods

### 2.1. Patient Clinical Information

A total of 312 patients who underwent hysteroscopic polypectomy of EP in our hospital from June 2017 to November 2020 were enrolled retrospectively. Inclusion criteria are as follows: (1) patients aged from 20 to 45 years old with EP underwent hysteroscopic polypectomy, and postoperative pathology showed endometrial polyps; (2) all patients were treated voluntarily; (3) there was no desire to have children within one year; (4) there was no abnormality in biochemical examinations and patients without acute reproductive tract infection or other contraindications for transvaginal operation; and (5) patients without uterine leiomyoma, endometriosis, polycystic ovary syndrome, and other gynecological benign and malignant diseases.

Exclusion criteria are as follows: (1) smokers; (2) thrombotic diseases, with a history of deep phlebitis or venous thromboembolism; (3) circulatory and cerebrovascular diseases; (4) benign and malignant tumors and liver function abnormalities such as cirrhosis or active hepatitis; (5) diabetes-related complications such as diabetic nephropathy and diabetic retinopathy; and (6) patients who failed to receive follow-up observation and whose data were incomplete and could not be statistically analyzed.

### 2.2. Treatment Method

Among the 312 patients in this study, there were 42 patients who did not take any treatment after the operation (control group), 156 patients who were treated with levonorgestrel intrauterine birth control system (Mirena group), and 114 patients who were treated with spironolone ethinylestradiol tablet (Yasmin) after the operation (oral group) (the age of patients in oral Yasmin group should be less than 40 years old.).

Hysteroscopic polypectomy of EP is as follows: all patients accepted blood routine examination, urine routine examination, stool routine examination, liver and kidney function test, electrolyte, blood coagulation function, infectious diseases, human chorionic gonadotropin, tumor markers, electrocardiogram, chest X-ray, uterine adnexal ultrasound, and other routine examination items. The gynecological examination was given, and the results showed that there was no obvious surgical contraindication. Except for the patients who needed emergency operation because of a large amount of vaginal bleeding, all the other patients underwent TCRP 3-7 days after menstruation. Vaginal irrigation and skin preparation were given before the operation. Misoprostol 0.4 mg was placed in the posterior vaginal fornix to soften the cervix in the evening or early morning before the operation. Fasting diet and eliminating related anesthesia taboos were done before the operation, and intravenous anesthesia or intravenous inhalation combined anesthesia was given. Using the hysteroscopic equipment produced by the Olympus or Stryker company, 5% mannitol solution or 0.9% normal saline was used as uterine dilation fluid, and the uterine dilation pressure was 80-100 mmHg, which should be adjusted according to the specific conditions during the operation. The patient emptied the bladder before the operation, took the bladder lithotomy position, and after the completion of anesthesia, routinely disinfected the towel, indwelled urinary catheterization, sterilized the vagina again, placed a vaginal endoscope to dilate the vagina and expose the cervix, clamped the cervical anterior lip with cervical forceps, and explored the depth of the uterine cavity with a probe. Uterine dilation sticks gradually dilated the cervix. After emptying the air bubbles in the intake pipe, the hysteroscope was placed, and the outlet valve was adjusted to make the field of vision clear. Carefully observe the condition of the cervical canal and the shape of the uterine cavity, check whether the uterine cavity was hyperemia, check the endometrial thickness and suspected endometrial malignant change, and observe the size, number, growth location, and root pedicle of polyps. Special attention should be paid to observing the uterine floor, bilateral uterine corners, and bilateral fallopian tube openings, and the cervix should be checked again when withdrawing from the hysteroscope. Patients with endometrial thickening or suspected endometrial diseases should be diagnosed and curetted first and sent for histopathological examination. Reenter hysteroscopy, and complete resection of EP under direct vision, mostly with circular electrodes; the depth of resection should not be too shallow or too much, and the an appropriate amount of the endometrium around polyps should be removed to reduce recurrence and wound electrocoagulation to stop bleeding. Finally, the condition of the uterine cavity was examined again to determine that the shape of the uterine cavity was normal, and there was no active bleeding after the application of antiadhesion drugs to end the operation. All the scraped intimal tissue and resected polyp tissue were sent to routine histopathological examination after being examined by the family members. After the operation, patients were routinely given appropriate fluid replacement, antibiotics to prevent infection, and other symptomatic treatment, and patients were advised to pay attention to rest, have no basin bath and sex life for 1 month, and keep the vulva clean and dry.

The control group is as follows: there was no special treatment except routine treatment after the operation.

The oral group is as follows: oral spironolone ethinylestradiol tablets (manufacturer: Bayer Pharmaceutical and Health Co., Ltd. Guangzhou Branch, approval number: J20130120, specification: each tablet contains spirosterone 3 mg and ethinylestradiol 0.03 mg 21 tablets/box, trade name: Yasmin) for 3 cycles immediately after the EP is confirmed by postoperative histopathological examination.

The Mirena group is as follows: the endometrial polyps are confirmed by postoperative histopathological examination to place levonorgestrel intrauterine birth control system (levonorgestrel-releasing intrauterine system, LNG-IUS, manufacturer: Bayer Medical and Health Co., Ltd. Guangzhou Branch, approval number: J20140088, specification: 52 mg/containing levonorgestrel, trade name: Mirena) on the 3rd-5th day after the first menstruation.

### 2.3. Observation Index

The clinical data of 312 patients were recorded and followed up regularly. All patients were followed up through an outpatient clinic or telephone to 12 months after the operation. The patients' age, course of the disease, number of pregnancies, clinical manifestations, endometrial thickness before the operation, duration of operation, amount of bleeding during the operation, and number and size of polyps were analyzed. Endometrial thickness, symptom improvement, and hemoglobin were followed up 3, 6, and 12 months after the operation. The recurrence and postoperative adverse reactions of EP in the three groups were followed up within 12 months after the operation.

Diagnostic criteria of recurrence of EP are as follows: postoperative color Doppler ultrasound showed suspicious signs of the endometrium such as endometrial thickening, uneven echo of the endometrium, or slightly higher echo of uterine cavity; patients with or without abdominal pain, abnormal vaginal bleeding, increased secretions, and other clinical manifestations, no taboo to give secondary surgical treatment, and confirmed by postoperative pathology as EP are defined as recurrence.

### 2.4. Statistical Method

The SPSS 20.0 statistical software was used to analyze the measurement data, and *t*-test was used to analyze the measurement data. For example, *n* (%) was used to represent the count data, *χ*^2^ test was adopted, and repeated measurement data were analyzed by repeated measures analysis of variance (ANOVA). The difference was statistically significant (*P* < 0.05). In addition, a *P* value less than 0.001 is viewed as highly statistically significant (*P* < 0.001).

## 3. Results

### 3.1. To Compare the General Condition and Operation of the Three Groups of Patients

There was no significant difference in age, course of disease, times of pregnancy, abnormal vaginal bleeding, number of polyps, diameter of polyps, intraoperative bleeding volume, and diagnostic curettage among the three groups (*P* > 0.05). All the results are indicated in Table 1.

### 3.2. The Thickness of the Endometrium and the Level of Hemoglobin Were Compared among the Three Groups

There was no significant difference in endometrial thickness among the three groups before treatment (*P* > 0.05). After 3, 6, and 12 months of treatment, the endometrial thickness of the three groups decreased, while the decrease in the Mirena group and the oral group was better compared to the control (*P* < 0.001). The decrease in the Mirena group was better than that in the oral group (*P* < 0.001). There was no significant difference in hemoglobin levels among the three groups before treatment (*P* > 0.05). After 3, 6, and 12 months of treatment, the hemoglobin levels of the three groups increased to varying degrees, while the levels of the Mirena group and oral group were better compared to the control (*P* < 0.001). The level of the Mirena group was higher than that of the oral group (*P* < 0.001). All the results are indicated in Table 2.

### 3.3. To Compare the Improvement of Clinical Symptoms among the Three Groups of Patients

After treatment, the symptoms of abdominal pain were relieved even disappeared, there was no abnormal vaginal bleeding or a reduced amount of bleeding, and no increase of vaginal secretions was regarded as an improvement of clinical symptoms. Follow-up and statistics were made on the improvement of clinical symptoms of patients in different groups at 3, 6, and 12 months after the operation.

Three months after the operation, among the 42 patients in the control group, 37 patients' clinical symptoms were improved, 5 patients' clinical symptoms were not improved, and the improvement rate was 88.09%. Among the 114 patients in the oral group, 102 patients had improvement in clinical symptoms, and 12 patients had no improvement in clinical symptoms. The improvement rate was 89.47%. Among the 156 cases in the Mirena group, 141 patients' clinical symptoms were improved, 15 patients' clinical symptoms were not improved, and the improvement rate was 90.38%. The improvement of clinical symptoms was similar among the three groups, and there was no significant difference among the three groups (*P* > 0.05).

Six months after the operation, 38 patients in the control group had clinical symptoms improved, 4 patients had no improvement in clinical symptoms, and the improvement rate was 90.47%. Among the 114 patients in the oral group, 107 patients had improvement in clinical symptoms, and 7 patients had no improvement in clinical symptoms. The improvement rate was 93.85%. Among the 156 patients in the Mirena group, 151 patients' clinical symptoms were improved, 5 patients' clinical symptoms were not improved, and the improvement rate was 96.79%. The improvement of clinical symptoms in the oral group and Mirena group was better than that in the control group (*P* < 0.05), but there was no significant difference between the oral group and Mirena group (*P* > 0.05).

Then, 12 months after the operation, the clinical symptoms of 33 patients in the control group were improved with a rate of improvement 78.57%; however, 9 patients had no improvement. Among the 114 patients in the oral group, 105 patients had improvement in clinical symptoms, and 9 patients had no improvement in clinical symptoms. The improvement rate was 92.11%. Among the 156 cases in the Mirena group, 150 patients had clinical symptoms improved, 6 patients had no improvement, and the improvement rate was 96.15%. The improvement of clinical symptoms in the oral group and Mirena group was better compared to the control (*P* < 0.05), and the improvement of clinical symptoms in the Mirena group was better than that in the oral group (*P* < 0.05).

### 3.4. Comparison of Complications and Recurrence among the Three Groups

After the operation, some patients had complications such as lower abdominal pain, breast distension pain, irregular vaginal bleeding, and abnormal liver function. There was no significant difference in the number of complications among the three groups (*P* > 0.05). During the follow-up to 12 months, the recurrence rate in the oral group and Mirena group was lower compared to the control (*P* < 0.05), and the recurrence rate in the Mirena group was lower than that in the oral group (*P* < 0.05). All the results are indicated in Table 3.

## 4. Discussion

EP remains one of the common diseases in gynecology, which has the characteristics of high incidence, diverse manifestations, less malignant transformation, easy recurrence, and so on [1]. Some studies have shown that the incidence of EP varies greatly according to the definition of polyps, the diagnostic methods used, and the groups studied, which is 7.8%-34.9% [20]. According to the literature, it is reported that the incidence of EP in postmenopausal women is the highest, about 31%. The peak age of endometrial polyps is at the age of 50, and EPs are more common in women over 35 years old, with an incidence of about 23% [21, 22]. The clinical manifestations of patients with EP are different, and the most common clinical manifestation is abnormal vaginal bleeding, which can be manifested in many ways, such as bleeding after the same room, intermenstrual bleeding, endless dripping after menstruation, frequent menstruation, and postmenopausal vaginal bleeding [21, 22]. In addition, EP is also one of the common causes of infertility in women of childbearing age. EP interferes with the implantation of fertilized eggs by affecting the shape of the uterine cavity, resulting in infertility or early abortion of women of childbearing age [23, 24]. Symptoms such as abdominal pain and increased vaginal secretions are also possible reasons for patients with EP. In recent years, with the continuous improvement of medical level, the diagnosis rate of some asymptomatic endometrial patients has also increased. Ultrasound is the most commonly used method to evaluate the condition of the endometrium, which can effectively diagnose parts of patients with EP. TVUS is the most commonly used way for the diagnosis of EP because of its advantages such as noninvasive, economical, and convenient operation, no need to prefill the bladder, avoiding the interference of abdominal fat layer and intestinal gas, and so on [7]. EPs have a large age range and a large number of patients, and most EPs are benign lesions. The American Association of Gynecologic Laparoscopy points out that 25% of EP can disappear on their own, especially those with a diameter less than 1 cm [25]. However, there are still a small number of endometrial malignant changes. A meta-analysis reported by Lee et al. showed that the rate of malignant transformation of endometrial polyps was 3.57% [26]. At present, hysteroscopic resection of EP combined with postoperative histopathological examination has become the gold standard for the diagnosis and treatment of EP. However, many scholars have not reached a consensus on the etiology and mechanism of EP, and EP is easy to recur after treatment. According to relevant literature, it is reported that whether patients are obese, the frequency of abortion, whether complicated with polycystic ovary syndrome, different postoperative treatment measures, the size of EP, whether complicated with abnormal uterine bleeding, follow-up time, and so on are the risk factors of EP recurrence [27]. In this study, we studied the endometrial thickness, symptom improvement, recurrence rate, and adverse reactions after hysteroscopic polypectomy. It is of important clinical value to explore how to scientifically and effectively reduce the recurrence of EP.

EP is a state of excessive hyperplasia of the endometrium, which is composed of endometrial glands, stroma, and locally hyperplastic blood vessels. Polyps vary in size, ranging from a few millimeters to a few centimeters in diameter, and the number of polyps varies from single polyps to multiple polyps [28]. With the increasing maturity of endoscopic technology, hysteroscopy has been widely used in the diagnosis and treatment of gynecological and obstetrical uterine diseases because of its direct vision, easy operation, less trauma, and quick recovery [29]. During hysteroscopy, we can directly observe the condition of the cervical canal and the shape of the uterine cavity, check whether the uterine cavity is congested and red, the thickness of the endometrium, and whether the endometrial malignant transformation is suspected, and observe the size, number, growth position and root pedicle of the polyp, the uterine floor, bilateral uterine horn, and bilateral fallopian tube opening [30].

At present, hysteroscopic resection of endometrial polyps combined with histopathological examination has become the primary choice for the diagnosis and treatment of EP. At present, most scholars believe that the disorder of estrogen and progesterone metabolism and the abnormal effect of estrogen and progesterone receptors in the endometrium may be the reason for the difference in the degree of intimal hyperplasia in different parts of the endometrium and the formation of polyps [31, 32]. ER and PR are expressed in endometrial glands and stroma and play a role by binding to estrogen and progesterone. Previous studies have shown that ER and PR are highly expressed in secretory endometrium. Estrogen may stimulate endometrial proliferation by promoting the synthesis of ER and PBR, while progesterone has the opposite effect [33]. The study on the expression levels of PR and ER in EP surrounding normal endometrium showed that the levels of ER and PR in endometrial polyps were significantly higher than that in surrounding normal endometrial cells, whether in glands or stroma, suggesting that the overexpression of ER and PR may play an important role in the pathophysiological process of polyps [34]. Overexpression of ER and PR, imbalance of estrogen and progesterone ratio, and use of estrogenic drugs were risk factors for endometrial polyps [35]. The expression levels of ER and PR were also related to the invasion and metastasis of endometrial carcinoma [36]. Therefore, the abnormal expression of ER and PR is closely related to the occurrence of EP, and improving this abnormal state may help to prevent the recurrence of EP.

Mirena is an intrauterine device containing levonorgestrel, which is T-shaped and covered with a special controlled release membrane, which can continuously and steadily release trace amounts of levonorgestrel (20 *μ*g/d) [37]. The concentration of progesterone released from the local endometrium is 1000 times higher than that of the plasma. It can directly act on the endometrium and glands, antagonize the stimulating effect of estrogen on the endometrium, induce the transformation of the endometrium to the secretory phase, make the glands atrophy and interstitial edema, lead to endometrial atrophy and decidua-like degeneration, and prevent the recurrence of endometrial polyps [37]. In addition, high levels of progesterone can also downregulate the immune activity of ER and PBR in endometrial glands and stroma, weaken the binding activity of estrogen and its receptor, reduce the sensitivity of the endometrium to circulating estrogen, avoid endometrial hyperplasia, and reduce EP recurrence [38].

In this study, the results showed that after 12 months of follow-up, the recurrence rate of EP decreased significantly, and it was more beneficial to improve the level of hemoglobin in patients. Because it can reduce menstruation and increase hemoglobin, the British NICE guidelines regard it as a first-line treatment for menorrhagia [39]. In addition, the follow-up of endometrial thickness also showed that the endometrium was significantly thinner in the Mirena group, suggesting that Mirena may inhibit endometrial hyperplasia and then prevent the recurrence of polyps. It should be pointed out that vaginal drip bleeding is a common adverse reaction after the placement of the Mirena, which may be due to the decrease of the level of PR, resulting in a decrease in the activity of progesterone-dependent prostaglandin dehydrogenase, resulting in increased vascular fragility [37]. It is related to bleeding, which can be relieved by itself and does not need special treatment.

In summary, placing Mirena immediately after hysteroscopic polypectomy of EP can reduce the recurrence rate of endometrial polyps, increase the level of hemoglobin, and reduce the thickness of the endometrium, which can be employed and popularized according to the condition of patients in clinical duties.

## Figures and Tables

**Table 1:** Comparison of general condition and operation among three groups of patients (*n* (%), $\bar{x}\pm s$).

Index	C group (*n* = 42)	Oral group (*n* = 114)	Man Yuele group (*n* = 156)	*F*/*χ*^2^	*P*
Age (years)	33.18 ± 5.28	32.78 ± 6.14	33.93 ± 5.77	1.311	0.271
Course of disease (month)	7.13 ± 2.28	6.92 ± 2.43	6.78 ± 2.55	0.357	0.700
Number of pregnancies (times)	2.57 ± 0.71	2.39 ± 0.62	2.44 ± 0.73	1.047	0.352
Abnormal vaginal bleeding					
Yes	23	60	79		
None	19	54	77	0.261	0.877
Number of polyps					
Single shot	17	51	72		
Multiple hair	25	63	84	0.433	0.805
Polyp diameter (cm)	2.24 ± 0.54	2.16 ± 0.83	2.21 ± 0.86	60.111	<0.001
Operation time (min)	29.58 ± 7.22	28.89 ± 7.35	29.21 ± 8.14	0.134	0.875
Intraoperative bleeding volume (ml)	8.56 ± 2.71	8.74 ± 2.51	8.61 ± 2.86	0.102	0.903
Diagnostic curettage					
Yes	21	55	74		
No	21	59	82	0.089	0.956

**Table 2:** Endometrial thickness and hemoglobin level in three groups of patients $\left(\bar{x}\pm s\right)$.

Group	*N*	Endometrial thickness (mm)				Hemoglobin level (g/l)			
		Before the operation	Three months after the operation	Six months after the operation	12 months after the operation	Before the operation	Three months after the operation	Six months after the operation	12 months after the operation
C group	42	12.65 ± 2.17	4.67 ± 1.01	6.25 ± 1.57	10.21 ± 2.06	105.39 ± 10.67	112.25 ± 12.71	118.39 ± 11.67	122.25 ± 13.78
Oral group	114	12.43 ± 2.35	4.48 ± 1.13	6.15 ± 1.45	8.29 ± 2.24	103.95 ± 11.48	116.87 ± 13.28	122.39 ± 12.47	125.25 ± 12.86
Man Yuele group	156	12.58 ± 2.25	3.48 ± 1.07	5.15 ± 1.38	6.29 ± 1.87	104.55 ± 11.27	120.87 ± 12.76	128.39 ± 12.65	132.25 ± 13.51
*t*		0.205	37.095	20.126	73.128	0.264	8.353	14.167	14.194
*P*		0.815	<0.001	<0.001	<0.001	0.768	<0.001	<0.001	<0.001

**Table 3:** complications and recurrence of patients in three groups (example, %).

Group	*N*	Occurrence of complications				Number of recurrent cases
		Dull pain in the lower abdomen	Breast pain	Irregular vaginal bleeding	Abnormal liver function	
C group	42	3 (7.14)	2 (4.76)	3 (7.14)	1 (2.38)	6 (14.28)
Oral group	114	7 (6.14)	5 (4.38)	6 (5.26)	3 (2.63)	6 (5.26)
Man Yuele group	156	12 (7.69)	7 (4.48)	11 (7.05)	10 (6.41)	4 (2.56)
*χ* ^2^		0.243	0.080	0.394	2.697	9.352
*P*		0.885	0.961	0.821	0.259	0.009

## Data Availability

No data were used to support this study.
